# Characterizations of infant flours and profiles of populations using them in the center of Côte d'Ivoire

**DOI:** 10.1016/j.heliyon.2024.e31644

**Published:** 2024-05-21

**Authors:** K.M. Gboko, K.Y. Koné, D. Soro, K.B. Yao

**Affiliations:** a Department of Chemical and Food Engineering, National Polytechnic Institute-HB, BP 1093, Yamoussoukro, Republic of Côte d'Ivoire; b African Center of Excellence for the Valorization of High Added Value Products, National Polytechnic Institute-HB, BP 1093, Yamoussoukro, Republic of Côte d'Ivoire

**Keywords:** Complementary foods, Infant flour, Malnutrition

## Abstract

**Introduction:**

Infant malnutrition is a public health issue observed in children from the age of 6 months, period of food diversification. The objective of this study was to characterize the infant flours intended for children from 6 to 24 months on the Ivorian market and to identify the profiles of the populations using them in order to improve a new type of flour manufacturing.

**Materials and methods:**

Then, a cross-sectional investigation was conducted among 300 households with young children in the center of Cote d'Ivoire. This survey should point out the different types of complementary foods percentages used in households and the ones who use these foods which have an impact on child malnutrition; this in order to highlight the social and economic factors which influence the practices of use, preferences and choices of complementary foods of the populations that use them.

**Results and discussions:**

The results indicate that 76 % of the households surveyed use industrial infant flours, 22 % traditional flours and 2 % make a combination of both industrial and traditional flours. The overall populations find imported manufactured flours too expensive with a preference rate of 41.5 %, 26 % for traditional flours and 32.5 % for products made up of the two previous ones. As for the practice of using complementary foods by households: 18 % practice it early, 54 % at the recommended age (6 months) and 28 % use them late.

**Conclusions:**

a preference for traditional flours by households is observed because of their accessibility (affordable prices). Also, to better the nutritional and economic qualities of these traditional flours would be a good strategy to fight against child malnutrition in Africa.

## 1 Introduction

Malnutrition is a global health issue which undermines the whole world [1]. This observation is aroused by the fact that populations adopt unbalanced and/or inadequate diets. This dietary imbalance creates an unfavorable nutritional status which is at odds with the reference values established by the reference organizations [2]. This fact is due to undernutrition, which is a deficiency in essential nutrients, or overeating, which is an excessive consumption of one or more nutrients essential to the proper functioning of the human metabolism.

In countries plagued by malnutrition, women and children are generally the most vulnerable [3].Then, when this malnutrition affects children, we refer then to it as infant malnutrition [2]. The recommendations of the WHO are such that, the child should be exclusively fed with breast milk until the age of six (6) months [4]. This recommendation unveils that, from six (6) months, breast milk is no longer sufficient to fulfill the nutritional needs of the child. Therefore, it is necessary to introduce complementary foods into the baby's diet [5].

In Africa, porridge is the most used food as supplement to breast milk in infant feeding [6]. That porridge is made of cereals and tubers that are high in carbohydrates but low in proteins [7]. Consequently, this porridge comes to fill in normal times, the lack of essential nutrients and the nutritional needs of the child from the age of six (6) months; what the mother's milk alone cannot provide in the child's diet [1]. This period of diversification of the infant's diet is very important for its health and proper development [8]. Thus, the products available on the local market are industrial flours which are either produced locally or imported [9]. These industrial flours relatively remain expensive and cannot be affordable to households, especially the low-income ones [10,11]. So, these ones run towards traditional flours which are much more accessible because of their low purchasing power [12]. However, the child's poor diet depends on many factors, ranging from the nutritional qualities of the complementary foods consumed [13], to the lack of knowledge of complementary foods, including bad practices related to the use of these products within infants' diet [14,15]..

From this observation, the practices for initiating the use of infant flours, the infant flours on the market and their nutritional and economic characteristics could have an influence on the choices for the purchase and use of complementary foods, hence their impact on child malnutrition in Côte d'Ivoire.

For the better formulations of infant flours based on local ingredients, it is necessary to know the nutritional and economic characteristics of the different flours of infant supplements that one can find on the local market. But it is also important to highlight the social and economic factors of the populations which influence the uses and the practices of introduction of the infant flours into the infant's diet.

This study aims at researching the infant flours intended for the complementary feeding of children from 6 to 24 months already on sale. It will also evaluate the profiles of the populations preferring these products and then, the social and economic causes which encourage their choice.

## 2 Materials and methods

### 2.1 Samples and areas of investigation

This survey is a cross-sectional study aimed at taking stock of infant flours intended for complementary feeding of children aged 6–24 months available for sale in Côte d'Ivoire, while also assessing the profiles of the populations using these products and the social and economic factors influencing their choices. The collection of socio-economic data for the study was carried out in Sakassou, which is a department in the Gbêkê region located in central Côte d'Ivoire. The department has a population of 69,386 inhabitants and 13,362 households with an average size of 5.2 persons [16]. Since the number of households with children under 5 years old is not known, it was assumed that 25 % of households have a child under 5 years old. Therefore, the sample size is determined using Schwartz's method based on the following formula:

$$N=\frac{t^{2}p\left(1-p\right)}{\varepsilon^{2}}$$

N: sample size; P: proportion of households with a child under 5 years (25 %); ε: absolute error risk of 0.05; t: 1.96 for a 95 % confidence level.

The obtained sample size is N = 288.12 households, which we round up to 300 households.

For the collection of nutritional data, the study focused on infant flours intended for children from six months to 24 months (2 years old), available and displayed in supermarkets in the city of Yamoussoukro located in central Côte d'Ivoire. The survey also took place in certain markets within the Yamoussoukro area, namely Djahakro, Assabou, and the main central market.

### 2.2 Data collection

The household survey involved 300 households residing in Sakassou and extended from August 4, 2022, to November 14, 2022. Recruitment was done through structured questionnaires featuring logos of participating institutions, aiming for completely voluntary participation of respondents through snowball sampling. Each household was individually visited for a semi-structured interview lasting approximately 30 min. To ensure participant anonymity, names and surnames were not requested but identified by order numbers.

For the collection of nutritional and economic data on infant complementary flours sold in Côte d'Ivoire, a second survey initially involved cataloging infant foods (infant flours) intended for children from six months to two years old. To compile this list, investigations were conducted in five (5) wholesale and semi-wholesale supermarkets in the city of Yamoussoukro, namely SOCCOCE, King Cash, Cash Ivoire, Super Mag, and CDCI. Additionally, certain online selling platforms (Jumia and Jumia Food) were also visited. Price data were obtained from displayed price labels in the supermarket aisles, while nutritional compositions were noted from information directly on the product packaging encountered in the retail outlets.

### 2.3 Inclusion and exclusion criteria

Inclusion criteria required being a parent of a child under 5 years old at the time of the survey and residing in the Sakassou department while voluntarily agreeing to answer questions during the interview. Exclusion criteria included refusal to participate in the interview and absence of children under 5 years old in the household.

### 2.4 The analysis results

The collected data analysis during the survey was carried out using GraphPad Prism 8 software (Dotmatics, Boston, Massachusetts). The comparisons of the means of the different parameters were carried out by the test of analysis of the variances with two factors (ANOVA 2-ways), the study of the correlations was carried out by the method of “R of Pearson”. The overall analyzes were performed with a margin of error of 5 % (α = 0.05).

## 3 Results

### 3.1 Characteristics of the different types of infant flours on the Ivorian market

#### 3.1.1 Typology and proportion of infant flours

The surveys conducted at the sales areas level in the department of Yamoussoukro, made it possible to identify twenty-seven (27) infant flours frequently present in the five (5) sales areas and online sales platforms (Table 1). Among these twenty-seven (27) infant flours, twenty-four (24) are produced by industrial companies and three (3) are manufactured through artisanal ways. Industrially produced flours are subdivided into two groups. The first group consists of products processed by companies established on the Ivorian territory. These firms are Nestlé, PKL les précuits and GLP les précuits. The second group consists of industrial products imported from the Blédina and France Lait companies (Table 1). Apart from industrial flours, there are flours traditionally produced by local populations based on corn, millet and rice flour.

**Table 1:** Type of infant flour available on the Ivorian market and their place of production and sales areas.

Type of Flour	Origin	Business	Infant Flours	Presence in Sales Areas
Industrial Infant Flours	Local	Nestlé	Cerelac wheat	(1), (2), (3), (4), (5), (6)
			Cerelac wheat with milk	(1), (2), (3), (4), (5), (6)
			Cerelac fruit-milk	(1), (2), (3), (4), (5), (6)
		PKL	Farinor apple nutribon	(1), (2), (3), (4), (5), (6)
			Farinor wheat soy milk	(1), (2), (3), (4), (5), (6)
			Farinor corn soy milk	(1), (2), (3), (4), (5), (6)
		GLP	Corn flour	(1), (3)
			Rice flour	(1), (3)
			Plain soy flour	(1), (3)
	Imported	Blédina	Blédina milk cereal bananas and milk	(1), (2), (3), (4), (5), (6)
			Blédina cereal milk wheat fruit	(1), (2), (3), (4), (5), (6)
			Blédina milky growth	(1), (2), (3), (4), (5), (6)
			Blédina milky fruits	(1), (2), (3), (4), (5), (6)
			Blédina milky honey	(1), (2), (3), (4), (5), (6)
			Blédina honey milk	(1), (2), (3), (4), (5), (6)
			Biscuit Milk Phosphatine	(1), (2), (3), (4), (5), (6)
			Milky Phosphatine Wheat	(1), (2), (3), (4), (5), (6)
			Phosphatine honey	(1), (2), (3), (4), (5), (6)
			Maize-Rice Milk Phosphatine	(1), (2), (3), (4), (5), (6)
		France milk	France Diastase milk	(1), (2), (3), (4), (5), (6)
			France milk wheat and honey	(1), (2), (3), (4), (5), (6)
			France milk wheat-fruit	(1), (2), (3), (4), (5), (6)
			France milk-rice-honey	(1), (2), (3), (4), (5), (6)
			France milk wheat-biscuit	(1), (2), (3), (4), (5), (6)
Traditional infant flours	Local	Anonymous	Millet flour	(7)
			Rice flour	(7)
			Corn flour	(7)

NB: the presence of a number opposite a product means that this product was present in the sales area corresponding to this number. (1): SOCCOCE, (2): King cash, (3): Cash Ivoire, (4): Super Mag; (5): CDCI; (6): Online sales platforms; (7): Local markets.

All of the industrial infant flours were found in all the sales areas, except for the flours produced by GLP (corn, rice and soya flours) which were only present in two sales areas. As for the local traditional infant flours were only found in one sales area.

#### 3.1.2 Classification of infant flours according to price

The price of infant flour found on the Ivorian market varies between 150 FCFA/500 g of the product (minimum price attributed to traditional maize flour) and 3719 FCFA/500 g (maximum price allotted to industrial flour) (Exp. Cerelac fruit and milk). The average cost of traditional flour is 163 ± 13 (FCFA/500 g). Therefore, the average cost of industrial flour is 2842 ± 351 (FCFA/500 g).

The comparison of the different prices by the analysis of variances to show a significant difference between those prices (Fig. 1) with a *p-value <0.05.* This difference allows the classification of these products into five (5) groups. In descending price order, the flour with the highest price is "Cerelac fruit" (3719 FCFA/500 g), followed by a group of Blédine products with an average price of 3332 ± 114 FCFA/500 g, then phosphatines and Blédina milk, wheat, and fruit flours of 2828 ± 94 FCFA/500). The fourth group is made up of “Farinor corn, soy, milk and Farinor wheat soy milk” flours, then “Cerelac wheat” flour with an average price of 2667 ± 111 (FCFA/500 g). The last group is that of traditional flours with the lowest average cost which is 163 ± 13 (FCFA/500 g).

**Fig. 1:** Price comparison chart for infant flours available on the Ivorian market. **NB**: The presence of the same lower-case letter above several bars indicates that there is no significant difference (p-value >0.05) between flour prices by comparison of variances in the AVOVA test. Otherwise, it indicates a significant difference (p-value <0.05), α = 0.05.

Flour prices are marked by differences, this could be due to the difference in the ingredients used for production. The fact that the unit operations for the transformation of the different ingredients into flour are not the same, could also influence the production costs of the flours; Unlike the flours produced traditionally, without formulation or complex production means, which are at a lower cost.

#### 3.1.3 Comparison of the nutritional compositions of infant flours with the standard

The data relating to the nutritional compositions acquired on the labels of infant flours underwent a two-factor analysis of variance (ANOVA) compared to the reference (standard) nutritional values.

The results of this analysis revealed that, there was no significant difference (p*-value* = 0.1743 and α = 0.05) between the nutritional values of infant flours available on the Ivorian market and the ones the *Codex- Alimentarius* sets (Table 2) when we consider the average nutritional values overall. However, by taking the components individually, one can see significant differences (with a *p-value <0.0001* and α = 0.05) between the different compared products. Thus, Infant flours have an energy value which generally varies between 145 and 439 ± 28.33 (Kcal) per 100 g of flour, 2.92 and 17.9 ± 3.3 (g) for proteins, 0.41 and 10 ± 2.82 (g) for lipids, 0.22 and 86 ± 12.78 (g) for carbohydrates, 0.1 and 5.7 ± 1.38 (g) for fibers, 0.3 and 53.3 ± 3.7 (mg) for vitamins and 1.2 and 228.1 ± 57.19 (mg) for minerals. Commercial brand flours such as Blédina, Cerelac and Farinor have energy values from 386 to 439 kcal per 100 g of product. Protein contents vary from 7.4 to 17.9 g, fat from 2 to 10 g and carbohydrates from 60 to 86 g. Traditional flours, made from millet, rice and maize, have respective energy values of 145, 456 and 346 kcal per 100 g of product. These flours are distinguished by their low protein (less than 3 g per 100 g), fat (less than 4 g) and fiber (less than 6 g per 100 g) content, while the carbohydrate content varies from 0.22 to 67.2g per 100g. The Pearson statistical test (with P = 0.0027; r = 0.5 and α=0,05), showed that there was a positive correlation between the average nutritional values and the prices of the flours available on the market (Fig. 2). Fig. 3 shows the correlation between the different groups of flour compounds.

**Table 2:** Comparison of nutritional values of weaning flours on the Ivorian market with WHO and *Codex Alimentarius Standards*.

**NB:** The red color represents the highest values and the blue color represents the lowest values in the same column.

**Fig. 2:** Scatter plot of the linear regression (The Pearson statistical test) of the average nutritional value of flours as a function of price.

**Fig. 3:** Correlation table of the nutritional value of flours as a function of price.

### 3.2 Profiles of households using infant flours

The household survey covered 300 people, including 78 men (26 %) and 222 women (74 %). 20 % of respondents were under 20, 42 % between 20 and 30, 28 % between 30 and 40, 4 % between 40 and 50 and 6 % over 50.

#### 3.2.1 Profession impacts on the profile of infant flour users

Fig. 4 provides information on the proportions of the populations surveyed in accordance with professions.

**Fig. 4:** Proportions of infant flour users in accordance with profession. NB: The presence of the same lower-case letter above several bars indicates that there is no statistically significant difference between them based on the ANOVA test. Otherwise, there is a significant difference. P < 0.0001; α = 0.05.

The results in Fig. 4 show a diversity of professions within the population sample surveyed. Shopkeepers and housewives represent the highest proportions, with respectively 16 % and 18 % of the sample. This testifies the importance of the commercial sector and domestic chores within this population. Pupils and students also represent significant proportions (8.5 % and 14 % respectively), which reflects the presence of an active school and university population. Teachers are another important category with 12 % of the sample, indicating the importance of education in this community. Among other represented professions, one can find workers such as pharmacy auxiliaries, electricians, masons, mechanics, carpenters, midwives and executive secretaries. Although these occupations have lower proportions, they nevertheless contribute to the diversity of professional skills noticed in the sample. It is necessary to notice that the relative proportions of occupations can vary across samples and specific contexts. The collected data in this study can provide useful information for understanding the socio-economic dynamics and occupational structures of this population.

During the analysis of Fig. 4, it comes out that the existence of a highly significant difference (p*<0.0001; α = 0.05)* between the proportions of the different professions; meaning that occupations strongly influence the profiles of infant flours users. However, there is no significant difference (P*=0.4915;* α = 0.05) between the proportions of farmers and executive secretaries. This means that these two professions have the same infant flours use profile.

Therefore, the most important populations who use infant flours are housewives and traders with respectively 18 % and 16 %. This stresses that these two segments of the population are more in contact with children and can be consulted for the implementation of a future formulation of infant flour. Then, come the students with 14 %, teachers with 12 % and pupils with 8.5 %, indicating that these fringes of intellectuals, more aware of the benefits of infant flour, should not be neglected in the process of planning a new infant flour.

As for the other segments of the surveyed population, they use infant flour in a small proportion: either for lack of time (with management secretaries (6 %), and pharmacy auxiliaries (1.5 %)); or because they consider them expensive (this is the case for farmers (6 %), carpenters (5 %), mechanics (4 %), masons (3 %) and electricians (2 %)).

The obtained results picture a distribution of children using infant flours according to different age groups. These data are represented by Fig. 5 in relation to the number of children encountered in households according to age groups from 0 to 7 years.

**Fig. 5:** Graph representing the age groups of the children of the surveyed families.

The surveyed households had children with an age range between one (1) and seven (7) years. 13.5 % of these children were aged between 0 and 1 months, 42 % between 1 and 2 months, 24.5 % between 2 and 3 months, 7 % between 3 and 4 months, 4 % between 4 and 5, 3 % between 5 and 6 months and 6 % between 6 and 7 months. The largest proportion of children encountered in households were between zero (0) and three (3) years old with a proportion of 80 %. Therefore, 20 % of these children were in an age group of three (3) to seven (7) years.

According to the data from the respondents (Fig. 6), 76 % of those questioned used industrial infant flours, 22 % used traditional infant flours and 2 % combined both industrial and traditional infant flours. This means that people are more aware of the benefits of industrial flours for their children, especially with the complementary foods they provide.

**Fig. 6:** Diagram representing the use proportions of infant flour types. **NB:** The presence of the same lowercase letter above several bars indicates that there is no statistically significant difference between them. Otherwise, it marks a significant difference. P < 0.0001; α = 0.05.

Fig. 7 presents the percentages of preferences for the use of different types of flour on the market by the surveyed populations. Overall, according to the surveys, infant flours are represented by 11 brands or combinations of brands used by the populations. Traditional infant flours are the most used with a proportion of 26 %. They are followed by "Blédine" brand flours with 23.5 %, "Cerelac" brand flours with 18 % and the combination of "Phosphatine + traditional flours" with 9 %.

**Fig. 7:** Use of infant flour by preference of the surveyed populations. **NB:***The different types of flour are represented on this graph by codes which are the first 4 letters of the trade name. Cerelac (Cere), Blédina (Bled), Nido growth (Nido), Blédilait (Blel), Phosphatine (Phos), Traditional flour (Trad), Mashed potatoes (Pomm), Francelait (Fran).*

The other flours have a lower percentage. These are "Phosphatine" flours which represent 5 %, the combination of "Cerelac + traditional flours + mashed potato" flours and "Blédilait" products representing 4 % each. Next come the “Nido Growth” brands with a percentage of 3.5 % and “Francelait” with a proportion of 3 %. Finally, come the brand combinations “Blédine + phosphatine” and “Blédine + phosphatine + Nido Growth” which have the lowest fractions of 2 % each.

### 3.3 Impacts of the economic income during the period of infant flours use

The periods of introduction of complementary foods in the diet of children in the surveyed households are displayed in Fig. 8.

**Fig. 8:** The age impact on the introduction of infant complementary foods into children's diets.

This graph shows that the surveyed households started using infant flours in the diet of children from the age of three months. 18 % of households introduced infant flours a little earlier before the recommended age of six months. However, 28 % of households introduced complementary flours into the children's diet later after the children were six (6) months old.

## 4 Discussions

The objective of this study was to establish the nutritional profiles of various infant flours designed for children aged 6–24 months available in the Ivorian market. Simultaneously, the study aimed to characterize the populations using these complementary foods and the socio-economic factors influencing their usage practices, with the goal of adding value to a future flour formulated from local ingredients.

Consequently, a survey identified 27 infant flours commonly used for the dietary supplementation of young children (6–24 months). Despite the availability of numerous raw materials and the potential to combine them to create infant formulae, 55.56 % of encountered manufactured products were imported, with 33.33 % produced locally, alongside 11.11 % traditional flours. This is likely attributed to Côte d'Ivoire not being an industrialized country. Additionally, it could be explained by the complexity of combining local ingredients due to the absence of technology and existing nutritional formulas for formulating infant flours using these available ingredients, or perhaps by inadequate awareness of these local resources as ingredients for complementary food formulation.

The results of this analysis demonstrate significant diversity in the nutritional composition of infant flours available in the Ivorian market. Industrial flours such as those from Blédina, Cerelac, and Phosphatine Lactée are generally high in energy (439 Kcal), protein (17.9 g/100g), and fat (10 g/100g), which aligns with the nutritional needs of growing infants. According to the WHO, good nutrition during infancy is crucial for physical and mental growth and development. Unfortunately, many infants do not receive balanced and regular diets, leading to malnutrition issues. The proliferation of processed foods can also contribute to dietary imbalances and reduced breastfeeding rates. Breastfeeding has been shown to be crucial for overall child development [17]. WHO collaborates with partners to promote optimal nutrition for infants and young children by encouraging breastfeeding and preventing malnutrition [18]. This variability in nutritional content may be due to the significant and varying number of ingredients used in formulating flour-based supplements. It may also be explained by the aim of fortifying specific nutrients, particularly vitamins and minerals, to promote proper child development. To prevent vitamin and mineral deficiencies and ensure a healthy intake of essential nutrients, food fortification should be guided by a fundamental principle of public health [19]. Fortifying wheat and maize flours, widely consumed staple foods processed centrally, could have a significant impact on micronutrient malnutrition. Fortification programs have the advantage of reaching large population groups through existing food distribution systems without requiring changes to current consumption standards [19]. The fortified elements differ depending on the ingredients used and the food production structure. However, there is no significant difference in the overall nutritional averages of the flours considered, as each formulation is carried out according to recommendations from national or international regulatory bodies. Nonetheless, traditional flours exhibit low nutritional quality compared to Codex Alimentarius recommendations [20]. These observations are consistent with those of [21], which indicate that porridge made from traditional maize, millet, or sorghum flour consumed by children has a relatively low energy density. In Burkina Faso, it ranges from 36 to 60 Cal/100 mL, in Gabon from 44 to 64 Cal/100 mL, and in Congo at 60 Cal/100 mL [19]. Moreover, simple cereals-based flours have low protein content, thus limiting the availability of essential amino acids like lysine and tryptophan, reflecting nutrient imbalances [22]. Furthermore, traditional millet, rice, and maize flours, although lower in calories and certain essential nutrients, are natural options that bring local flavors and richness in specific fibers and minerals [23]. They can complement industrial flours by providing dietary variety and cultural adaptation in infant feeding [[24], [25], [26]].

A positive correlation has been established between the price and the average nutritional value of infant flours. The higher the nutritional value of a product, the more expensive it tends to be. This suggests that the nutritional value of flours depends on the quality and cost of the ingredients used, as well as the production processes involved in making these flours. For the same production unit, there is no significant difference in prices among products with similar average nutritional qualities. A likely reason for this is the use of identical equipment and processes. As a result, traditional flours are cheaper with lower average nutritional values compared to standard values [27].

Analysis of the population profile by age reveals a low proportion of respondents under 20 years old, as most individuals in this age group are typically students without children and dependent on their parents. The majority of respondents aged 20–40 years old represent the working-age population. Additionally, those surveyed in this age group generally have some form of regular income, enabling them to support themselves and manage a household. Furthermore, a significant number of homemakers (18 %) and artisans (16 %) were surveyed. Homemakers are prevalent in households due to their daily activities, while artisans are found in shops and workshops near households, making them easily accessible. Surveys were conducted on weekdays. Students rank second (14 %) as they comprise civil servants or financially independent individuals with children. Traders, being an important professional group, have easier access to various brands of infant flour and can choose from a variety of options based on their preferences and income. Students and teachers, representing a substantial proportion, may opt for infant flours due to convenience and ease of use. Homemakers, representing the largest proportion, play a crucial role in feeding infants and young children. Their choice to use infant flours may be influenced by factors such as availability, ease of use, and confidence in product quality [28,29]. It is noteworthy that certain professions, such as pharmacy assistants, midwives, and executive secretaries, are also involved in using infant flours. These healthcare and medical professionals may be more aware of the importance of infant nutrition and recommend specific flours based on infants' needs. Despite a high rate (22 %) of industrial infant flour usage, all respondents stated that the selling prices of these products were high. Additionally, once prepared, these flours are difficult to store as they lose consistency and become liquid. Consequently, individuals with limited financial means have started feeding their children industrial complementary foods combined with traditional flours such as cornmeal, millet flour, rice porridge, and mashed potatoes. As a result, another portion of this population sticks to using traditional complementary foods due to limited means. Those using industrial infant preparations generally have some level of education and perceive industrial products as higher quality. Moreover, some rely on these industrial flours based on recommendations from healthcare professionals (midwives, nurses, or doctors). Traditional infant flours are most commonly used by the poorest populations. Additionally, illiterate individuals prefer these traditional flours out of ignorance, believing they have similar nutritional qualities to industrial products. However, slightly literate populations with some knowledge of the nutritional benefits of manufactured products, despite their limited means, combine manufactured and traditional products. Intellectual households, with financial means and awareness of the benefits of complementary foods (from manufactured products), exclusively use industrial infant flours.

The analysis of data based on children's ages reveals interesting trends regarding the use of infant flours. Children under one year old, representing a significant proportion, are particularly reliant on infant flours for their nutrition, as they still have specific nutritional needs. Infant flours are often used as a supplement to breastfeeding or as a substitute when breastfeeding is not possible. As children grow older, their dependence on infant flours gradually decreases. Children aged 1–2 years represent the largest proportion, which can be attributed to the transition from breastfeeding or infant flours to complementary feeding. Infant flours can help provide the necessary nutrients at this crucial stage of child development. It is noteworthy that even after the age of 2 years, a significant proportion of children continue to use infant flours. This may be due to individual preferences, established habits, or specific needs related to certain health issues or nutritional deficiencies.

The data analysis highlights a dominant trend of introducing infant flours predominantly from the age of 6 months. Among those who used infant flours (Fig. 6), 54 % started complementary feeding in addition to breast milk (maternal or manufactured) from 6 months onwards, considering exclusive milk feeding to be insufficient for the child's nutritional needs. This trend is consistent with international and national recommendations on infant feeding, advocating for the introduction of complementary foods, including infant flours, from the age of 6 months while continuing breastfeeding [17,30]. Similar practices were observed in a study in Benin, where 64 % of mothers introduced complementary foods from 6 months, which is the ideal time. It is important to note that 18 % of surveyed families started using infant preparations slightly earlier, from the age of 3 months. This practice may be attributed to individual factors such as specific nutritional needs or issues with insufficient breastfeeding or availability [5].

The reasons given by mothers of these children were that they did not have enough breast milk to adequately feed the child or they did not have enough time to breastfeed due to work or illness. These same observations, with similar justifications, were made in a survey on infant porridge by Ref. [5]. In this study, it was found that 73.33 % of the surveyed mothers practiced early introduction of complementary foods into the baby's diet. It also happens that the reason for this early use of infant complementary foods is that the child is not consuming breast milk. This is a risky practice because it is important to emphasize that exclusive breastfeeding is recommended until the age of 6 months to meet the nutritional and immunological needs of infants [31]. Indeed, children under 4 months of age may not have developed physiology to digest foods other than breast milk. Additionally, breast milk covers most of the body's water needs for the child. Therefore, early weaning could lead to dehydration and even expose the child to potential deficiencies in essential fatty acids (EFAs), iron, and calcium [32]. The proportions of introducing infant flours at 4 months (10 %) and 5 months (6 %) also indicate variations in feeding practices. Some families may choose to introduce infant flours a little earlier for various reasons, such as the child's gradual adaptation to different textures or individual food preferences. The last group, comprising the smallest proportions at ages 7 months, 8 months, and 9 months (10 %, 8 %, and 8 % respectively), can be attributed to a gradual transition to more solid and diversified food, where infant flours may be supplemented with other foods such as fruits, vegetables, and unprocessed cereals. This group started complementary feeding later, after the child reached six months of age. Individuals in this group believed it was better to prolong exclusive breastfeeding a little longer, which is incorrect as breast milk alone is not sufficient to meet the child's nutritional needs during this period. Another reason is based on financial constraints, according to data collected during the survey. However, delayed introduction of complementary foods reduces the child's tolerance window to allergens between 4 and 6 months [33]. Therefore, these children are more likely to develop food allergies. Early contact (between 5 and 6 months) with allergens progressively and incrementally would allow the child's body to accept them as non-allergens [34].

### 4.1 Strengths and limitations of the study

The study on the use of complementary foods in central Côte d'Ivoire presents several significant strengths. Firstly, it addresses a relevant issue concerning food security and nutrition in a region where these issues are critical. The adopted methodology allows for detailed data collection on family eating habits, thereby providing a wealth of information for policymakers and public health stakeholders. Additionally, the study highlights socio-economic factors that influence the choice of complementary foods, which can guide targeted policy development. However, the study also has limitations. It should be noted that this study is one of the first conducted in this part of Côte d'Ivoire on complementary foods. Thus, the geographical scope limited to a single department of the region may not reflect the diversity of eating practices across the entire Ivorian territory. Similarly, the results could be influenced by seasonal biases, as food access may vary throughout the year. It is also possible that self-reported data from participants may not be entirely reliable, which could affect the accuracy of the conclusions. Lastly, the study could benefit from comparative analysis with other regions to better contextualize its findings. In summary, although the study makes important contributions to understanding the use of complementary foods in central Côte d'Ivoire, it should be considered within the framework of its methodological and geographical limitations. Further research would be needed to confirm and extend its findings to a broader context.

## 5 Conclusions

This study has allowed to make an assessment of the different infant flours intended for children from 6 to 24 months. It was found that 74 % of infant flours come from manufactured and imported products with a high purchase price. However, the 26 % of traditional infant flours made from local cereals (corn, rice and millet), although less expensive, are not rich in nutritional value.

The results of the surveys indicate that overall, the populations are aware of the need for the use of infant food supplements, but the financial means would hinder the proper use of these foods. Therefore, it is necessary to produce accessible infant food supplements to all social classes while respecting the recommendations of regulatory bodies.

Relying on these data, a preference for traditional flours by households is observed because of their accessibility. However, it is agreed that an improvement in the nutritional qualities and economic aspects of these flours could be a good strategy for weaning children and fighting against the child malnutrition.

## Funding statement

This work was supported by the Africa Center of Excellence for Waste Valorization into High Value-Added Products (CEA-ValoPro).

## Data availability statement

The data used are included in the article.

## Declaration of ethics

As the author of this study on the “characterisation of infant formula and profiles of the populations using it in central Côte d’Ivoire”, I would like to emphasize the fundamental importance of ethics in the conduct of our research. Our commitment to scientific integrity, respect for human rights and transparency guides every aspect of this study. This survey was previously authorised by the prefect of the Sakassou department before data collection.

Informed consent: All participants in this socio-economic survey were fully informed of the objectives of the research, the procedures involved and their rights as participants. Informed consent was obtained voluntarily and documented. Participants were assured of the anonymity of their responses and the confidentiality of their data.

## Ethical approval

This study was conducted in strict accordance with the ethical standards established by the Polytechnic Doctoral School (EDP). The committee evaluated and approved our research protocol, thereby ensuring that all activities carried out were ethical and respectful of participants’ rights.

Confidentiality of data: All information collected has been treated as confidential. The data are stored securely and will only be accessible to members of the research team. The results presented in this manuscript do not allow individual identification of participants.

Respect for the populations studied: We recognise the diversity and richness of the cultures in Côte d’Ivoire. Interactions with participants were conducted with the greatest respect for their traditions, customs and values.

Transparency and scientific integrity: We are committed to reporting the results of our research in a transparent manner, whether they confirm or refute our initial hypotheses. No intentional bias has been introduced into the collection, analysis or presentation of the data.

This ethics statement demonstrates our commitment to conducting responsible and respectful research, contributing to the advancement of knowledge while honouring the rights and dignity of the individuals who participated in our study.

Approved by: Prof. Dr. YAO Kouassi Benjamin, Director of the Polytechnic Doctoral School; Senior Lecturer, Dr. KONE Kisselmina Youssouf, Thesis Director; Senior Lecturer, Dr. SORO Doudjo, Thesis Director.

## CRediT authorship contribution statement

**K.M. Gboko:** Writing – original draft, Methodology, Investigation, Formal analysis, Data curation, Conceptualization. **K.Y. Kone:** Writing – review & editing, Validation, Supervision. **D. Soro:** Writing – review & editing, Validation, Supervision. **K.B. Yao:** Supervision.

## Declaration of generative AI and AI-assisted technologies in the writing process

During the preparation of this work, the author used Deepl in order to reformulate certain content for a better understanding of the information. After using this tool, the author reviewed and edited the content as needed and take full responsibility for the content of the publication.

## Declaration of competing interest

The authors declare that they have no known competing financial interests or personal relationships that could have appeared to influence the work reported in this paper.
